This article has been retracted.

# Serum sTREM-1 and CXCL-16 Levels in Children with *Mycoplasma pneumoniae* Pneumonia and Their Diagnostic Value

**DOI:** 10.1155/2021/7179796

**Published:** 2021-10-13

**Authors:** Chengchao Fang, Yueyan Mao, Mingfen Jiang, Wei Yin

**Affiliations:** ^1^Department of Pediatrics, The First People's Hospital of Yuhang, Yuhang District, Hangzhou, Zhejiang 311100, China; ^2^Department of Hemodialysis Center, The First People's Hospital of Yuhang, Yuhang District, Hangzhou, Zhejiang 311100, China

## Abstract

*Mycoplasma pneumoniae* pneumonia (MPP) is an acute respiratory tract infection caused by *Mycoplasma pneumoniae*. It is characterized by severe symptoms, long course of disease, many intrapulmonary complications, and poor therapeutic effect. In recent years, the incidence of *Mycoplasma* infection have been gradually rising trend, and the children's own immune system development is not mature, cases differences, children with mild can only show the upper respiratory tract infection, and critically ill children can lead to lung infection and even lead to multiple organ dysfunction, affect life and health of children. Soluble triggering receptors expressed on myeloid cell-1 (sTREM-1) is a subtype secreted by myeloid cell trigger receptor-1, which is released into blood in large amounts when the body is infected, and is a newly discovered inflammatory indicator in recent years. CXC chemokine 16 (CXCL-16) can recruit lymphocytes by chemotaxis through binding to its receptor CXCR6 to participate in the body's immune regulation. The purpose of this study was to investigate serum sTREM-1 and CXCL-16 levels in children with MPP and to analyze their correlation with the disease and diagnostic value. The results showed that the serum levels of sTREM-1 and CXCL-16 were increased in children with *Mycoplasma*. Serum levels of sTREM-1 and CXCL-16 were positively correlated with the severity of the disease. sTREM-1 combined with CXCL-16 has an important value in the diagnosis of children with MPP.

## 1. Introduction

Pneumonia is one of the common pediatric diseases and the primary cause of death of hospitalized children in China [1, 2]. *Streptococcus pneumoniae*, *Mycoplasma pneumoniae*, and respiratory syncytial virus are the most common pathogens of infection [3, 4]. *Mycoplasma pneumoniae* pneumonia (MPP) is an acute respiratory infection caused by *Mycoplasma pneumoniae*, accounting for 10–30% of bronchopneumonia [5, 6]. In recent years, the incidence of *Mycoplasma* infection have been gradually rising trend, and the children's own immune system development is not mature, cases differences, children with mild can only show the upper respiratory tract infection, and critically ill children can lead to lung infection, and even lead to multiple organ dysfunction, serious life and health of children [7, 8]. There are many methods for diagnosis of MPP infection, among which the isolation and culture of *Mycoplasma pneumoniae* is a reliable standard for diagnosis of MPP infection. However, it takes a long time to culture, and the rapid culture is of limited value because of its low sensitivity and specificity, so it has little significance for early clinical diagnosis [9, 10]. Nucleic acid diagnostic technology has strong specificity, high sensitivity, and rapid and can be used for early diagnosis, but the technical requirements are high, and it is easy to be affected by the carrying state after MPP infection, so it is also not applicable to clinical practice [2, 11]. At present, methods such as lung X-rays and detection of *Mycoplasma* IgM antibodies are often used in clinical practice. Although the accuracy is high, it does not effectively reflect the severity of the disease. Therefore, it is extremely important to find specific indicators that can effectively reflect the severity of children with MPP and to screen critically ill children as soon as possible. Soluble triggering receptors expressed on myeloid cell-1 (sTREM-1) are an important inflammatory factor and index of oxidative stress. The increase of its concentration can lead to the activation of downstream inflammatory signaling pathways, improve the upregulation of effector factors such as interleukin-6, and cooperate with toll-like receptors to mediate the expansion of inflammatory response, thus promoting the progression of pulmonary infectious disease [12–14]. Among many chemokines and chemokine receptors, CXC chemokine ligand receptor-16 (CXCL-16)/CXCR6 is a pair of chemokine ligand-receptor pairs with unique functions. They are widely involved in many pathological and physiological processes, including lymphocyte recruitment, organ development, chronic inflammation, and cell survival. CXCL-16 can bind to its receptor CXCR6 to participate in the migration and adhesion of inflammatory factors to mediate the inflammatory response [15, 16]. The purpose of this study was to investigate serum sTREM-1 and CXCL-16 levels in children with MPP and to analyze their correlation with the disease and diagnostic value. The specific report is as follows.

## 2. Materials and Methods

### 2.1. Patients

64 children with MPP diagnosed in our hospital from March 2017 to September 2019 were selected as the observation group. Among them, 38 were males and 26 were females, aged 2–12 years old, with an average age of 6.86 ± 2.61 years old. Inclusion criteria: all met the diagnostic criteria for MPP [17]; no glucocorticoids and other immunosuppressive agents have been used in the past month; and clinical data are complete. Exclusion criteria: bronchopneumonia caused by other pathogens; patients with pulmonary tuberculosis and other lung diseases; patients with immune system diseases; and patients with malignant tumors. According to the clinical manifestations of the children, the observation group was divided into the following two subgroups. Mild group (*n* = 36): no oxygen inhalation or other auxiliary respiratory therapy was needed, the symptoms were mild, no large shadow was found on X-ray, and little or no rales of dry or wet were heard in the lungs. Severe group (*n* = 28): required oxygen inhalation and other auxiliary respiratory treatments, X-rays had large shadows, a lot of dry and wet rales could be heard in the lungs, and pulmonary complications such as pleural effusion and bronchiectasis occurred. 50 healthy children who underwent physical examination during the same period were selected as the control group. Among them, 29 were males and 21 were females, aged 1–12 years, with an average age of 6.34 ± 2.96 years old. There was no statistically significant difference between the two groups of gender and age in general data (*P* > 0.05), and they were comparable. This study was approved by the ethics committee of our hospital, and the patients and family members gave informed consent and signed an informed consent form.

### 2.2. Research Method

After admission, 4 ml of fasting venous blood was drawn from the two groups of children in the morning for testing. Serum levels of sTREM-1 and CXCL-16 were determined by the enzyme-linked immunosorbent assay (ELISA). The relevant test kits were purchased from Shanghai Yanyu Biotechnology Co., Ltd., and the specific operation methods were strictly in accordance with the instructions. The clinical pulmonary infection score (CPIS score) was used to assess the severity of the child's condition, with a maximum score of 12 points. The higher the score, the more severe the child's condition.

### 2.3. Statistical Method

The results of this experiment were statistically analyzed by SPSS 20.0 (SPSS Co., Ltd., Chicago, USA). Measurement data were expressed by mean ± standard deviation, and the *t* test was used for their comparison between groups. Pearson correlation analysis was used for correlation analysis. ROC curve was used to analyze the differential diagnostic value of sTREM-1 and CXCL-16 levels in children with *Mycoplasma* pneumonia. *P* < 0.05 indicates that the difference is statistically significant.

## 3. Results

### 3.1. Comparison of Serum sTREM-1 and CXCL-16 Levels between the Two Groups

Serum levels of sTREM-1 and CXCL-16 in the observation group were higher than those in the control group (*P* < 0.05), as shown in Figure 1.

### 3.2. Comparison of Serum sTREM-1 and CXCL-16 Levels in Children with Different Disease Severity

The levels of serum sTREM-1 and CXCL-16 in the severe group were higher than those in the mild group (*P* < 0.05), as shown in Figure 2.

### 3.3. Correlation between Serum sTREM-1 and CXCL-16 Levels in Children with Disease

Pearson correlation analysis showed that serum sTREM-1 and CXCL-16 levels were positively correlated with their disease (CPIS score) (*r* = 0.907, *r* = 0.892, *P* < 0.001), as shown in Figure 3.

### 3.4. Diagnostic Value of Serum sTREM-1 and CXCL-16 in Children with MPP

The area under the curve (AUC) of serum sTREM-1 for predicting prognosis in children with MPP was 0.742 (95% CI: 0.592–0.893). When the best cutoff value was 53.84 pg/mL and Youden index was 0.473, the sensitivity and specificity were 62.5% and 84.8%. The area under the curve (AUC) of serum CXCL-16 for predicting the prognosis of children with MPP was 0.696 (95% CI: 0.544–0.848). When the best cutoff value was 1.64 ng/mL and Youden index was 0.381, the sensitivity and specificity were 56.4% and 81.8%. The combined area under the curve (AUC) for predicting the prognosis of children with MPP was 0.866 (95% CI: 0.755–0.976). When the Youden index was 0.710, the sensitivity was 87.5% and the specificity was 83.5%, as given in Table 1 and Figure 4.

## 4. Discussion

MPP is the smallest pathogenic organism capable of living independently on a cell-free culture medium between the size of the bacterium and the virus. It causes respiratory diseases in children, including pharyngitis, bronchitis, and pneumonia. It also causes airway hyperresponsiveness, including asthma, as well as numerous extrapulmonary manifestations [18, 19]. *Mycoplasma pneumoniae* can enter the body through the respiratory tract through contact infection and then grow between ciliated epithelia, inhibiting ciliated activity and destroying epithelial cells to cause local tissue damage, thus causing MPP [20, 21]. MPP is a common respiratory tract infectious disease in pediatrics. Most of the cases are mild and have a good prognosis. However, in recent years, the reports of severe cases of *Mycoplasma* pneumonia have gradually increased. Its pathogenesis may involve many aspects, such as children of large ring lactone class antibiotic resistance, excessive immune inflammatory response, diagnostic delays, and mixed infection [22, 23]. Clinical symptoms are often characterized by severe symptoms, long course of disease, many internal and external pulmonary complications, and poor therapeutic effect, and sequelae such as atelectasis, bronchiectasis obliterans, bronchiolitis obliterans, and other sequelae can be left, which have a serious impact on the physical and mental health of children [24, 25]. In recent years, with the emergence of resistant strains, the originally effective antimicrobial effect is reduced and even invalid, coupled with the combination of factors such as bacteria, virus infection, eventually making MPP for the development of severe MPP, severe MPP progress is fast, easy to merge pulmonary complications, both inside and outside of clinical treatment is difficult, mortality is higher, there are a lot of bad effects on children's health growth. Therefore, early diagnosis and timely treatment of *Mycoplasma* pneumonia are very important in clinics.

Chemokines play an important role in the regulation of tumor cell proliferation, invasion, and metastasis and are involved in the development of inflammatory response [26, 27]. According to the position of the first two cysteine amino acids at the amino terminus, it can be divided into C, CXC, CC, and CX3C. CXCL-16 has two forms: binding and secretion. Secreted CXCL-16 can promote the growth of tumor cells by activating phosphatidylinositol 3-kinase/protein kinase B (P13K/Akt) signaling pathway through CXCL-16/CXCR6 axis and has chemotactic and recruitment effects on lymphocytes [28]. CXCL-16 is the only ligand of CXCR6 discovered so far. Although it belongs to the CXC chemotactic factor family, the structure of CXCL-16 has very unique characteristics. It is composed of four parts: chemotactic structure region, mucin stalk structure region, transmembrane structure region, and cytoplasmic structure region. CXCL-16 can be expressed in dendritic cells, macrophages, endothelial cells, smooth muscle cells, human early pregnancy trophoblast cells, and other cells and play a variety of biological regulatory roles through CXCR6.

In the process of exploring the pathogenesis of *Mycoplasma* pneumonia in children, it can be found that the changes of inflammation-related factors play an important role in promoting the spread of pulmonary infectious disease. sTREM-1 is a subtype of receptor-1 secreted by myeloid cells, which is released into the blood in large quantities when the body is infected, and is a newly discovered inflammatory indicator in recent years [29, 30]. Related studies have pointed out that the level of sTREM-1 can reflect the degree of infection of the body. When the infection is severe, the level of sTREM-1 will increase significantly. When the inflammation of the body is effectively controlled, the level of serum sTREM-1 will decrease [31]. Velásquez et al. believe that under the action of macrophages and neutrophils, the expression level of serum sTREM-1 will increase significantly and play a role in amplifying the inflammatory cascade [32]. sTREM-1 is an important chemokine and inflammatory factor, which can promote the activation of downstream inflammatory cascade factors through the activation of MAPK, and aggravate the spread of infectious diseases in the lung.

In the process of lung inflammation, sTREM-1 is an indispensable regulator. In normal lung tissues, sTREM-1 is selectively expressed by pathogen-clearing alveolar macrophages and is upregulated in the presence of bacteria and fungi [33, 34]. Studies have shown that the expression level of sTREM-1 in bronchial lavage fluid of patients with community-acquired pneumonia and hospital-acquired pneumonia is significantly higher than that of healthy controls. In addition, the level of sTREM-1 is correlated with the positive rate of blood culture and sputum culture in patients with community-acquired pneumonia, indicating that serum sTREM-1 can be used as an independent inflammatory indicator of pneumonia [34, 35]. CXCL-16 can chemotactically recruit lymphocytes by binding to its receptor CXCR6 to participate in the body's immune regulation [36]. The results of this study showed that the serum levels of sTREM-1 and CXCL-16 in the observation group were higher than those in the control group, and the levels of serum sTREM-1 and CXCL-16 in the severe group were higher than those in the mild group. It shows that the levels of serum sTREM-1 and CXCL-16 in children with *Mycoplasma* pneumonia are increased, and the levels of serum sTREM-1 and CXCL-16 are closely related to the condition of children with *Mycoplasma* pneumonia. The reason is that *Mycoplasma pneumoniae* can adsorb on the surface of respiratory epithelial cells of the host after entering the body, destroy the epithelial cells, and cause local tissue damage [37, 38]. It can also cause the body's oral immunity and the high expression of lymphocytes in the lungs, thus leading to the increase of serum sTREM-1 and CXCL-16 levels. Moreover, the results showed that the serum levels of sTREM-1 and CXCL-16 in children with *Mycoplasma* pneumonia were positively correlated with their illness (CPIS score), which further indicated that the serum levels of sTREM-1 and CXCL-16 were closely correlated with the illness of children with *Mycoplasma* pneumonia. With the increase of serum sTREM-1 and CXCL-16 levels, the children's condition became more serious.

ROC curve results showed that the AUC of serum sTREM-1 and CXCL-16 in the diagnosis of MPP was 0.742 and 0.696, respectively, and the combined AUC of sTREM-1 and CXCL-16 in the diagnosis of MPP was 0.866. The results show that the value of sTREM-1 combined with CXCL-16 in the diagnosis of MPP in children is significantly higher than that of a single test and has a higher diagnostic value. The detection of sTREM-1 combined with CXCL-16 in children with MPP can promptly assess the condition, which can help improve the prognosis of the children.

## 5. Conclusion

In summary, the levels of serum sTREM-1 and CXCL-16 in children with MPP are elevated. Serum levels of sTREM-1 and CXCL-16 were positively correlated with the severity of the disease. sTREM-1 combined with CXCL-16 has an important value in the diagnosis children with MPP and is worth of promotion.

## Figures and Tables

**Figure 1:** Comparison of serum sTREM-1 and CXCL-16 levels between the two groups. (a) Serum sTREM-1 levels in the two groups. (b) Serum CXCL-16 levels in the two groups. Compared with the control group, ^*∗*^*P* < 0.05.

**Figure 2:** Comparison of serum sTREM-1 and CXCL-16 levels in children with different disease severities. (a) Serum sTREM-1 levels in children with different disease severities. (b) Serum CXCL-16 levels in children with different disease severities. Compared with the mild group, ^*∗*^*P* < 0.05.

**Figure 3:** Correlation between serum sTREM-1 and CXCL-16 levels in children with disease. (a) Correlation between serum the sTREM-1 level and disease condition in children. (b) Correlation between the serum CXCL-16 level and disease condition in children.

**Figure 4:** Diagnostic value of serum sTREM-1 and CXCL-16 in children with MPP. (a) Diagnostic value of serum sTREM-1 in children with MPP. (b) Diagnostic value of serum CXCL-16 in children with MPP. (c) Diagnostic value of combined detection of serum sTREM-1 and CXCL-16 in children with MPP.

**Table 1:** Diagnostic value of serum sTREM-1 and CXCL-16 in children with MPP.

Predictive indexes	AUC	95% CI	Youden index	Sensitivity (%)	Specificity (%)	Cutoff value
sTREM-1	0.742	0.592–0.893	0.473	62.5	84.8	53.84 pg/mL
CXCL-16	0.696	0.544–0.848	0.381	56.4	81.8	1.64 ng/mL
Combined predictive	0.866	0.755–0.976	0.710	87.5	83.5	—

## Data Availability

The datasets used and analyzed during the current study are available from the corresponding author upon request.

## References

[1] Krafft C., Christy C. (2020). Mycoplasma pneumonia in children and adolescents. *Pediatrics in Review*.

[2] Jin X., Zou Y., Zhai J., Liu J., Huang B. (2018). Refractory *Mycoplasma pneumoniae* pneumonia with concomitant acute cerebral infarction in a child: a case report and literature review. *Medicine*.

[3] Lin M., Shi L., Huang A., Liang D., Ge L., Jin Y. (2019). Efficacy of levofloxacin on macrolide-unresponsive and corticosteroid-resistant refractory *Mycoplasma pneumoniae* pneumonia in children. *Annals of Palliative Medicine*.

[4] Li Q., Li Z. Y., Zhang J. (2019). Xiyanping plus azithromycin chemotherapy in pediatric patients with *Mycoplasma pneumoniae* pneumonia: a systematic review and meta-analysis of efficacy and safety. *Evidence-Based Complementary and Alternative Medicine*.

[5] Jujaray D., Juan L. Z., Shrestha S., Ballgobin A. (2018). Pattern and significance of asymptomatic elevation of liver enzymes in mycoplasma pneumonia in children. *Clinical Pediatrics*.

[6] Sondergaard M. J., Friis M. B., Hansen D. S., Jorgensen I. M. (2018). Clinical manifestations in infants and children with *Mycoplasma pneumoniae* infection. *PLoS One*.

[7] Narita M. (2010). Pathogenesis of extrapulmonary manifestations of *Mycoplasma pneumoniae* infection with special reference to pneumonia. *Journal of Infection and Chemotherapy*.

[8] Zeng W.-Y., Li Y., Xu Z.-L., Xie X.-L., Xu F.-Q., Rui N. (2018). Severe Mycoplasma pneumonia in child with bilateral parapneumonic effusion successfully treated with integrated Chinese and western medicine: a case report. *Chinese Journal of Integrative Medicine*.

[9] Rogozinski L. E., Alverson B. K., Biondi E. A. (2017). Diagnosis and treatment of *Mycoplasma pneumoniae* in children. *Minerva Pediatrica*.

[10] Medjo B., Atanaskovic-Markovic M., Radic S., Nikolic D., Lukac M., Djukic S. (2014). *Mycoplasma pneumoniae* as a causative agent of community-acquired pneumonia in children: clinical features and laboratory diagnosis. *Italian Journal of Pediatrics*.

[11] Biondi E., McCulloh R., Alverson B., Klein A., Dixon A., Ralston S. (2014). Treatment of mycoplasma pneumonia: a systematic review. *Pediatrics*.

[12] Zhao X., Xu L., Yang Z. (2020). Significance of sTREM-1 in early prediction of ventilator-associated pneumonia in neonates: a single-center, prospective, observational study. *BMC Infectious Diseases*.

[13] Zhang H. F., Zhang X., Sha Y. X. (2020). Value of sTREM-1 in serum and bronchoalveolar lavage fluid, apache II score, and SOFA score in evaluating the conditions and prognosis of children with severe pneumonia. *Chinese Journal of Contemporary Pediatrics*.

[14] Palazzo S. J., Simpson T. A., Simmons J. M., Schnapp L. M. (2012). Soluble triggering receptor expressed on myeloid cells-1 (sTREM-1) as a diagnostic marker of ventilator-associated pneumonia. *Respiratory Care*.

[15] Gough P. J., Garton K. J., Wille P. T., Rychlewski M., Dempsey P. J., Raines E. W. (2004). A disintegrin and metalloproteinase 10-mediated cleavage and shedding regulates the cell surface expression of CXC chemokine ligand 16. *The Journal of Immunology*.

[16] Hara T., Katakai T., Lee J.-H. (2006). A transmembrane chemokine, CXC chemokine ligand 16, expressed by lymph node fibroblastic reticular cells has the potential to regulate *T* cell migration and adhesion. *International Immunology*.

[17] Atkinson T. P., Balish M. F., Waites K. B. (2008). Epidemiology, clinical manifestations, pathogenesis and laboratory detection of *Mycoplasma pneumoniae* infections. *FEMS Microbiology Reviews*.

[18] Lee K. Y., Youn Y. S., Lee J. W., Kang J. H. (2010). *Mycoplasma pneumoniae* pneumonia, bacterial pneumonia and viral pneumonia. *Jornal de Pediatria*.

[19] Izumikawa K., Izumikawa K., Takazono T. (2014). Clinical features, risk factors and treatment of fulminant *Mycoplasma pneumoniae* pneumonia: a review of the Japanese literature. *Journal of Infection and Chemotherapy*.

[20] Tomaino J., Keegan T., Miloh T. (2012). Stevens-Johnson syndrome after mycoplasma pneumonia infection in pediatric post-liver transplant recipient: case report and review of the literature. *Pediatric Transplantation*.

[21] Saraya T., Watanabe T., Tsukahara Y. (2017). The correlation between chest X-ray scores and the clinical findings in children and adults with *Mycoplasma pneumoniae* pneumonia. *Internal Medicine*.

[22] Wang Chun K., See Wan Y., Poon Chuen W. (2016). Transient presence of lupus anticoagulant associated with mycoplasma pneumonia. *Asian Cardiovascular & Thoracic Annals*.

[23] Ding L., Zhao Y., Li X. (2020). Early diagnosis and appropriate respiratory support for *Mycoplasma pneumoniae* pneumonia associated acute respiratory distress syndrome in young and adult patients: a case series from two centers. *BMC Infectious Diseases*.

[24] She D. Y. (2021). Focus on the difficulties and challenges in the diagnosis and treatment of *Mycoplasma pneumoniae* pneumonia. *Chinese Journal of Tuberculosis and Respiratory Diseases*.

[25] Al Yazidi L. S., Hameed H., Kesson A., Herath A., Pandit C., Britton P. (2019). A 6-year-old girl with severe, focal *Mycoplasma pneumoniae* pneumonia. *Journal of Paediatrics and Child Health*.

[26] Shimaoka T., Nakayama T., Kume N. (2003). Cutting edge: SR-PSOX/CXC chemokine ligand 16 mediates bacterial phagocytosis by APCs through its chemokine domain. *The Journal of Immunology*.

[27] Ribeiro S. M. T. L., Lopes L. R., Costa G. d. P. (2017). CXCL-16, IL-17, and bone morphogenetic protein 2 (BMP-2) are associated with overweight and obesity conditions in middle-aged and elderly women. *Immunity & Ageing*.

[28] Steffen S., Abraham S., Herbig M. (2018). Toll-like receptor-mediated upregulation of CXCL16 in psoriasis orchestrates neutrophil activation. *Journal of Investigative Dermatology*.

[29] Tan J., Huang X., Wu M. (2020). Value of soluble triggering receptor expression on myeloid cells-1 level of alveolar fluid in early diagnosis of ventilator-associated pneumonia: a meta-analysis. *Chinese Critical Care Medicine*.

[30] Li C., Zhu L., Gong X. (2019). Soluble triggering receptor expressed on myeloid cells-1 as a useful biomarker for diagnosing ventilator-associated pneumonia after congenital cardiac surgery in children. *Experimental and Therapeutic Medicine*.

[31] Oudhuis G. J., Beuving J., Bergmans D. (2009). Soluble triggering receptor expressed on myeloid cells-1 in bronchoalveolar lavage fluid is not predictive for ventilator-associated pneumonia. *Intensive Care Medicine*.

[32] Velásquez S., Matute J. D., Gámez L. Y. (2013). Characterization of nCD64 expression in neutrophils and levels of s-TREM-1 and HMGB-1 in patients with suspected infection admitted in an emergency department. *Biomedica: Revista del Instituto Nacional de Salud*.

[33] Wang Y., Zhang S., Li L., Xie J. (2019). The usefulness of serum procalcitonin, C-reactive protein, soluble triggering receptor expressed on myeloid cells 1 and clinical pulmonary infection score for evaluation of severity and prognosis of community-acquired pneumonia in elderly patients. *Archives of Gerontology and Geriatrics*.

[34] Xie J., Zhang X. H., Zhu W. Y. (2015). Values for serum procalcitonin, C-reactive protein, and soluble triggering receptor expressed on myeloid cells-1 in predicting survival of patients with early-onset stroke-associated pneumonia. *Genetics and Molecular Research*.

[35] Matsuno A. K., Carlotti A. P. (2013). Role of soluble triggering receptor expressed on myeloid cells-1 for diagnosing ventilator-associated pneumonia after cardiac surgery: an observational study. *BMC Cardiovascular Disorders*.

[36] Weseslindtner L., Görzer I., Küng E. (2014). High CXCL-16 levels correlate with symptomatic disease in lung transplant recipients with human cytomegalovirus replication in the allograft. *American Journal of Transplantation*.

[37] Grover V., Pantelidis P., Soni N. (2014). A biomarker panel (bioscore) incorporating monocytic surface and soluble TREM-1 has high discriminative value for ventilator-associated pneumonia: a prospective observational study. *PLoS One*.

[38] Zhang Y., Mei S., Zhou Y. (2017). TIPE2 negatively regulates mycoplasma pneumonia-triggered immune response via MAPK signaling pathway. *Scientific Reports*.

